# Rapid Detection of Beta-Lactamases Genes among *Enterobacterales* in Urine Samples by Using Real-Time PCR

**DOI:** 10.1155/2022/8612933

**Published:** 2022-08-08

**Authors:** Mariem Yengui, Rahma Trabelsi, Lamia Khannous, Nour Elhouda Mathlouthi, Mohd Adnan, Arif Jamal Siddiqui, Emira Noumi, Mejdi Snoussi, Radhouane Gdoura

**Affiliations:** ^1^Research Laboratory of Environmental Toxicology-Microbiology and Health (LR17ES06), Faculty of Sciences, University of Sfax, Tunisia; ^2^Department of Biology, College of Science, Hail University, P.O. Box 2440, Hail 81451, Saudi Arabia; ^3^Laboratory of BioResources: Integrative Biology and Recovery, High Institute of Biotechnology-University of Monastir, Monastir 5000, Tunisia; ^4^Laboratory of Genetics, Biodiversity and Valorisation of BioResources, High Institute of Biotechnology-University of Monastir, Monastir 5000, Tunisia

## Abstract

The objective of this study was to develop and evaluate newly improved, rapid, and reliable strategies based on real-time PCR to detect the most frequent beta-lactamase genes recorded in clinical *Enterobacterales* strains, particularly in Tunisia (*bla_SHV12_*, *bla_TEM_*, *bla_CTX-M-15_*, *bla_CTX-M-9_*, *bla_CMY-2_*, *bla_OXA-48_*, *bla_NDM-1_*, and *bla_IMP_*) directly from the urine. Following the design of primers for a specific gene pool and their validation, a series of real-time PCR reactions were performed to detect these genes in 78 urine samples showing high antibiotic resistance after culture and susceptibility testing. Assays were applied to DNA extracted from cultured bacteria and collected urine. qPCR results were compared for phenotypic sensitivity. qPCR results were similar regardless of whether cultures or urine were collected, with 100% sensitivity and specificity. Out of 78 multiresistant uropathogenic, strains of *Enterobacterales* (44 *E. coli* and 34 *K. pneumoniae* strains) show the presence of the genes of the *bla* group. In all, 44% *E. coli* and 36 of *K. pneumoniae* clinical strains harbored the *bla* group genes with 36.4%, 52.3%, 70.5%, 68.2%, 18.2%, and 4.5% of *E. coli* having *bla_SHV-12_*, *bla_TEM_*, *bla_CTX-M 15_*, *bla_CTX-M-9_*, *bla_CMY-2_*, and *bla_OXA-48_* group genes, respectively, whereas 52.9%, 67.6%, 76.5%, 35.5%, 61.8, 14.7, and 1.28% of *K. pneumoniae* had *bla_SHV-12_*, *bla_TEM_*, *bla_CTX-M 15_*, *bla_CTX-M-9_*, *bla_CMY-2_*, *bla_OXA-48_*, and *bla_NDM-1_* group genes, respectively. The time required to have a result was 3 hours by real-time PCR and 2 to 3 days by the conventional method. Resistance genes of Gram-negative bacteria in urine, as well as cultured bacteria, were rapidly detected using qPCR techniques. These techniques will be used as rapid and cost-effective methods in the laboratory. Therefore, this test could be a good candidate to create real-time PCR kits for the detection of resistance genes directly from urine in clinical or epidemiological settings.

## 1. Introduction

Urinary tract infections (UTIs) are among the most common infectious diseases in humans and represent a real public health problem in terms of both their frequency and their difficulty of treatment. *Enterobacterales* is primarily responsible for UTIs. *Escherichia coli* is the main pathogen responsible for cystitis and pyelonephritis as well as other species of *Enterobacterales*, such as *Proteus mirabilis* and especially *Klebsiella pneumoniae* [1, 2].

*Β*eta-lactams are the antibiotics preferentially used against these *Enterobacterales*. The emergence and spread of these bacteria producing extended-spectrum *β*-lactamases (ESBLs) or carbapenemases, have become a concern. In fact, the increase in the number of strains expressing *β*-lactamases (*E. coli*, *K. pneumoniae*) might be explained by the massive use of broad-spectrum cephalosporins (third-generation cephalosporins: C3G and fourth-generation cephalosporins: C4G). Moreover, this selection pressure adhered to the broadening of the TEM and SHV spectrum (by mutation of the *bla_TEM-1_* and *bla_SHV-1_* genes) and to the emergence of the CTX-M family, capable of hydrolyzing the penicillins, broad-spectrum cephalosporins, and aztreonam [3].

The dissemination of CTX-Ms enzymes has resulted in a generalization of their distribution throughout the world [4]. They are now the most extensively ESBLs in the world where the most common mutants are CTX-M-15 and CTX-M-14 belonging, respectively, to the CTX-M-1 and CTX-M-9 groups [5]. In Africa and Europe, recent studies have found a substantial increase in ESBL-producing Gram-negative bacteria causing community urinary tract infections, particularly harboring the *bla_CTX-M-15_* allele [6, 7].

Furthermore, over the last two decades, extended-spectrum *β*-lactamase (ESBL) and plasmid-mediated AmpC- (pAmpC-) producing *Enterobacterales* exhibiting resistance to the 3GCs has been increasingly isolated in humans [8]. Among the *AmpC β*-lactamase genes, particularly *bla_CMY-2_* and *bla_DHA-1_* are the most common in *E. coli* and *K. pneumoniae* strains, respectively, of human and companion animal [9, 10].

On the other hand, additional enzymes called carbapenemases have been detected in *E. coli* and *K. pneumoniae* strains. The OXA-1 type enzymes are sometimes hosted alongside the CTX-M group exhibiting ESBL activity, and class D *β*-lactamases hydrolyzing carbapenems (for example OXA-23, OXA-24/40, OXA-48, OXA-51, and OXA-58) are commonly found in *Pseudomonas aeruginosa* and *Acinetobacter baumannii* [11, 12].

As elsewhere in the world, the spread of multidrug-resistant (MDR) *E. coli*, often ST131, complicates treatment and attributes to massive use of previously reserved antibiotics, such as carbapenems and colistin [13]. One potential way to address these issues is to switch from empirical therapy to early-targeted therapy, detecting antibiotic resistance genes directly from clinical samples, with no culture that can take 2 to 3 days to become available. This identification can be achieved by metagenomic sequencing [14] although there is skepticism about the implementation, depending on costs and workflows [15]. The polymerase chain reaction (PCR) system was more immediately deployable, was less expensive, and has been frequently studied for proliferate mecA or carbapenemase genes, making it easier to treat infections [16, 17].

For this reason, our work is aimed at developing a qPCR system for the detection of *bla_TEM_*, *bla_SHV-12_*, *bla_CTX-M-15_*, *bla_CTX-M-9_*, *bla_CMY-2_*, *bla_OXA-48_*, *bla_IMP-1_*, and *bla_NDM-1_* group genes directly from urines and applying it in clinical *E. coli* and *K. pneumoniae* strains. An alternative to its methods through PCR can reduce the wait time to just a few hours.

## 2. Materials and Methods

### 2.1. Microbial Study

During the study period from December 2018 to December 2020, 2000 urine samples were collected from patients aged 20 to 65 years. Five hundred of them were culturally positive. Urine samples were collected from patients in health facilities as well as community patients in the towns of Sfax, south of Tunisia. All the strains collected were identified using the API 20E system (bioMérieux SA, Marcy l'Etoile, France).

#### 2.1.1. Phenotypic Characterization

Urine analysis and strain identification were performed by conventional methods. Antimicrobial susceptibility study was determined using the standard disk diffusion method on Mueller Agar-Hinton (Oxoid) according to Clinical Laboratory Guidelines and Institute Standards [18]. Tested antibiotics (Bio-Rad) were as follows: amoxicillin-clavulanate, (10 *μ*g) (AMX); amoxicillin, (20 *μ*g/10 *μ*g) (AMC); cefotaxime, (30 *μ*g) (CTX); ceftazidime, (30 *μ*g) (CAZ); cefoxitin (30 *μ*g) (FOX); amikacin (30 *μ*g) (AN); ciprofloxacin (10 *μ*g) (CIP); nalidixic acid (10 *μ*g) (NA); gentamicin (10 *μ*g) (GEN); netilmicin (30 *μ*g) (NET); tobramycin (10 *μ*g) (NN); fosfomycine (10 *μ*g) (FFL); trimethoprim + sulfamide (10 *μ*g) (SXT); imipenem (10 *μ*g) (IPM); and colistin (10 *μ*g) (CL). The diameters of the zones of inhibition were interpreted according to the recommendations of the CLSI [18]. All strains isolated were screened for extended-spectrum *β*-lactamase (ESBL) production by the double-disk synergy test [19].

### 2.2. Molecular Methods

#### 2.2.1. DNA Extraction

The DNA template was prepared according to a previously reported method with some modification [20, 21]. A loop of bacteria colonies harvested from a McConkey agar plate was suspended in 250 *μ*l of sterile distilled water and heated at 100°C for 10 minutes. After centrifugation at 15000 rpm for 5 min, the supernatant containing the harvested DNA was collected and stored at -20°C until its use in the PCR experiments.

The preparation of the DNA template from urine samples was conducted as follows: the urine (4–10 ml) was centrifuged at 12,000 rpm for 10 min, with the resulting bacterial pellet resuspended in 100 *μ*l of PVG and treated with an ADNucleis extraction and purification kit (ADNucleis, veterinary diagnostic platform, Lyon, France), for the lysis of the bacterial cells and to eliminate their DNA. Bacterial lysis buffer, lyophilized enzyme powder (PE), and enzyme mix suspension buffer (TME) were added, and after incubation for 10 min at 58°C, the DNA was purified using the BM Nucleic Acid Isolation Kit Based on Magnetic Beads [22].

#### 2.2.2. Primer Design

Based on the literature, primer design was performed using the BLAST (English Basic Local Alignment Search Tool) program to detect *β*-lactamase genes encoding extended-spectrum *β*-lactamases (*bla_SHV-12_*, *bla_TEM_*, and *bla_CTX-M-15_*) [23], Plasmid-mediated AmpC-lactamases (*bla*_CMY-2_) [24], and classes B (*bla_IMP-1_*, *bla_NDM-1_*) and D (*bla_OXA-48_*) carbapenemases [25]. These primers were verified by Primer 3 (Table 1).

#### 2.2.3. Real-Time PCR Amplification Program

The qPCR assay was performed on a CFX96™ real-time PCR thermocycler (BioRad, France).

Each reaction was carried out in a 20 *μ*l reaction mixture containing 1 *μ*l of template AND extracted directly from urine or from strains (50 ng/*μ*l), 100 nM of each primer, and 10 *μ*l of the SYBR green.

The optimal program of the qPCR includes an initial denaturation at 95°C for 3 min, followed by 40 cycles of: 95°C for 10 s; a hybridization temperature of 56°C for the genes *bla_TEM_*, *bla_SHV-12_*, *bla_CTX-M-15_*, *bla_CTX-M-9_*, and *bla_CMY-2_* and 60°C for the genes of group *bla_OXA-48_*, *bla_IMP-1_*, and *bla_NDM-1_* for 10 s and 72°C for 30 s. A melting step was performed at the end of the amplification; it was performed using the following cycling parameters: 60°C for 30 s and 5°C temperature changes to the end temperature of 95°C. The amount of amplified product was monitored by detecting the fluorescence energy emitted by SYBR green. Each PCR run included a negative control (no template control).

### 2.3. Determination of Specificity and Sensitivity of the qPCR Using Cultured Bacteria or Bacteria Harvested from Urine

Specificity and sensitivity were determined using the following formula: specificity = (*D*/*C* + *D*) × 100 and sensitivity = (*A*/*A* + *B*) × 100, where *A* is true positive, *B* is false negative, *C* is false positive, and *D* is true negative (Table 2). The values of the correlation coefficients *R*^2^ were calculated by the standard curve method. These values (*R*^2^) were 0.98 for all genes.

### 2.4. Statistical Analysis

Statistical tests including the *χ*^2^ test, multivariate logistic regression analysis to interpret the associations between the genes of the bla group and the different levels of antibiotic resistance, OR, and 95% CI were calculated as well as the analysis of Spearman's rank correlation. A *p* value of 0.05 was counted as statistically significant in this study. All data was done using IBM SPSS version 21.0.

## 3. Results

Of the 500 positive urine cultures, only the most predominant isolates were isolated, and among them, 90 isolates were considered multidrug-resistant strains, as these isolates were found to be resistant to at least two classes of antibiotics. Forty-four strains were identified as *E. coli*, which was predominant, followed by 34 strains of *K. pneumoniae*, 3 strains of *Enterobacter cloacae*, 2 strains of *Pseudomonas aeruginosa*, 2 strains of *Enterococcus faecalis*, 1 strain of *Morganella morganii*, 1 strain of *Citrobacter koseri*, 1 strain of *Aeromonas hydrophila*, 1 strain of *Acinetobacter*, and 1 strain of *Staphylococcus aureus.*

The qPCR system was used for the detection of antimicrobial resistance genes (Tables 2 and 3) in 78 uropathogenic *Enterobacterales* strains (44 strains of *E. coli* and 34 strains of *K. pneumoniae* included 40 strains of *E. coli* and 20 strains of *K. pneumoniae* ESBL producers), regardless of whether the DNA was extracted from bacteria in culture, or directly from urine.

qPCR reactions were initially performed at different annealing temperatures designated for each primer pair (Table 1).

### 3.1. Evaluation of Specificity and Sensitivity of the qPCR Using Cultured Bacteria or Bacteria Harvested from Urine

The newly developed qPCR system was effective in detecting genes of the *bla* group. The use of this system has shown that all the *Enterobacterales* isolates tested have at least one gene of the *bla* group. Of these, 31 contained more than three genes from the *bla* group. qPCR amplification of DNA extracted directly from urine was also performed. A concordance of 100% was found between the results of resistance genes detected directly from urine to those using purely isolated colonies (Table 2).

For the targeted *bla* group genes, the specificity and sensitivity of qPCR were both determined to be 100%.

### 3.2. Distribution of the Types blaSHV, blaTEM, blaCTX-M-15, blaCTX-M-9, blaCMY-2, blaOXA-48, blaNDM-1, and blaIMP-1 Group Genes in Clinical Enterobacterales Strains

qPCR data show that among the *E. coli* clinical strains, group genes *bla_CTX-M-15_* (70.5%, 31 strains), *bla_CTX-M-9_* (68.2%, 30 strains), bla_TEM_ (52.3%, 23 strains), and *bla_SHV-12_* (34%, 16 strains) were the most prevalent followed by group genes *bla_CMY-2_* (18.2%, 8 strains) and *bla_OXA-48_* (4.54%, 2 strains). None of these stains show the presence of the genes of the group *bla_NDM-1_* and *bla_IMP-1_*.

In *K. pneumoniae*, *bla_CTX-M-15_* (76.5%, 26 strains) was the most detected followed by *bla_SHV-12_* (52.9%, 18 strains), *bla_TEM_* (67.6%, 23 strains), *bla_CMY-2_* (61.8%, 21 strains), *bla_CTX-M-9_* (35.3%, 12 strains), *bla_OXA-48_* (14.7%, 5 strains), and *bla_NDM1_* (2.9%, 1 strains) group genes (Figure 1).

In addition, we found that 98.7% (*n* = 77) of the clinical *E. coli* and *K. pneumoniae* strains tested had at least one gene from the *bla* group with up to 34 different *bla* genotypes.

Otherwise, 25 (56.8%) of *E. coli* and 23 (61.5%) of *K. pneumoniae* had more than 2 genes. The most frequent combinations of 3 or more genes from the *bla* group of isolates tested have been summarized in Table 3.

### 3.3. Antibiotic Resistance Rates of the Clinical Enterobacterales Strains

The antimicrobial susceptibility testing performed for 78 *Enterobacterales* isolates (44 *E. coli* and 34 *K. pneumoniae*) showed that 60 (90.9%) of isolates were ESBL producers (40 *E. coli* and 20 *K. pneumoniae*).

Multidrug-resistant *E. coli* and *K. pneumoniae* strains show strong resistance to penicillin-family antibiotics such as amoxicillin, amoxicillin-clavulanate, ticarcillin, and 3rd-generation cephalosporin antibiotics such as cefotaxime and ceftazidime.

According to the test of the sensitivity of multiresistant *E. coli*, a high level of resistance was also recorded to ofloxacin, ciprofloxacin and nalidixic acid with a percentage of 95.5%, 93.2% (% CI [81.34% -98.57%]), and 88.6% (% CI [75.44% -96.20%]), respectively. Strains of *K. pneumoniae* also showed a high level of resistance to ofloxacin 85.3% (% CI [68.94% -95.04%]), ciprofloxacin 82.4% (% CI [65.46% -93.23%]), and nalidixic acid 85.3% (% CI [68.94% -95.04%]). A relative low resistance was recorded for imipenem with a percentage of 2.3% for *E. coli* and 29.4% (% CI [15.09% -47.47%]) for *K. pneumoniae*.

Otherwise, resistance to cefoxitin can also be considered to be low in strains of *E. coli* and *K. pneumoniae* with a percentage of 9.1% (% CI [2.53%-21.66%]) and 41.2 (% CI [24.64% -59.30%]), respectively. Clinical strains of *E. coli* were also resistant to other non-*β*-lactam antibiotics such as netilmicin 59.1% (% CI [43.24% -73.66%]), gentamicin 45.5% (% CI [30.39% -61.15%]), tobramycin 63.6% (% CI [47.77% -77.59%]), amikacin 25% (% CI [13.19% -40.33%]), bactrim 68.2% (% CI [52.42% -81.39%]), and fosfomycin 9.1% (% CI [2.53%-21.66%]). In addition, the 34 strains of *K. pneumoniae* showed resistance to netilmicin, gentamicin, tobramycin, amikacin, bactrim, and fosfomycin with a percentage of 52.9% (% CI [35.12% -70.22%]), 61.8% (% CI [43.56% -77.83%]), 61.8% (% CI [43.56% -77.83%]), 17.6% (% CI [6.76% -34.53%]), 67.6% (% CI [49.47% -82.61%]), and 50% (% CI [32.42% -67.57%]), respectively. None of these strains shows resistance to colistin (Table 4).

### 3.4. Relationship between Genotypic and Phenotypic Results of Resistance of Strains to Antibiotics

qPCR was carried out for the 78 uropathogenic strains of *Enterobacteriaceae* (44 E. coli and 34 *K. pneumoniae*) to analyze the ESBL genes as well as the determinants of resistance to drugs conferring resistance to *β*-lactam. The detailed associations of drug resistance with bla group detected in *K. pneumoniae* and *E. coli* isolates have been summarized in supplement Tables 5–7).

Resistance to four or more *β*-lactam antibiotics was associated with the presence of four genes from the bla group. Indeed, the analysis of the present data using the chi-square test showed a highly significant correlation between the resistance to four or more -lactams and blaTEM (*P* value = 0.006), blaCTX-M9 (*P* value = 0.008), and blaOXA-48 (*P* value = 0.006) (Table 5). Many strains harboring the blaTEM genes have also cohosted the genes of the blaCTX-M-9 groups. This positive association between the gene(s) of the blaTEM and/or blaCTX-M-9 group and resistance to four or more antibiotics was confirmed by multiple logistic regression analysis (Table 6) and by Spearman's rank correlation analysis (Table 7). In addition, a positive correlation was also recorded between the blaCMY-2 gene and the agent FOX. This association was proved by the chi-square test (*P* < 0.001; Table 5), multiple logistic regression (*P* = 0.002; Table 6), and Spearman's rank correlation analysis (*P* < 0.001; Table 7).

## 4. Discussion

qPCR system is a faster and more efficient technology for detection sensitivity to antibiotics compared to classical phenotypic and conventional methods [26]. It has been widely used for the research of resistance genes in clinical samples, but principally to support infection controlling rather than guiding therapy [21]. We explored its potential to detect important genes for antibioresistance to *Enterobacterales* in the clinic urine without culture.

Unlike most tests currently available (conventional methods), our qPCR system offers the advantage of detecting the target group of 7 *bla* genes (*bla_SHV_*, *bla_TEM_*, *bla_CTX-M-1_*, *bla_CTX-M-9_*, *bla_CMY-2_*, *bla_OXA-48_*, and *bla_NDM_*) after 2 hours with similar sensitivity and specificity which was obtained for both urine and cultured bacteria. For this reason, the detection of antibioresistance genes directly from biological samples could be a useful tool in Tunisia and other countries where the bla_CTX-M_ gene clusters were predominant. The CTX-M, TEM, and SHV enzymes were among the most common variants in Tunisia [27], in Palestine, in Egypt [28], and in European region [29] with varying prevalence rates. These results are similar to our qPCR data. Among the clinical strains of *E. coli*, *bla_CTX-M-15_* (70.5%) and *bla_CTX-M-9_* (68.2%) group genes were the most prevalent followed by *bla_TEM_* (52.3%), *bla_SHV_* (36.4%), *bla_CMY-2_* (18.2%), and *bla_OXA-48_ (*4.5%) group genes. In *K. pneumonia* strains, *bla_CTX-M-15_* (85.3%) was the most detected followed by *bla_SHV-12_* group (52.9%), *bla_TEM_* (67.6%), *bla_CMY-2_* (61.2%), *bla_CTX-M-9_* (35.3%), *bla_OXA-48_* (14.7%), and *bla_NDM-1_* (2.9%) group genes.

The qPCR test achieves a sensitivity of 100% and 100% specificity of the *β*-lactamase genes in clinical urine and cultured strains. Our results are in agreement with those of Schmidt et al. [14] who developed a multiplex tandem PCR (MT-PCR) for the detection of 16 genes of the ESBLs family in clinical urine and isolates cultured with a sensitivity of 100% and a specificity of 95-100% [30].

Uniformly, these results using urine directly are comparable to that proven by others using analogous methodology on cultivated isolates. Chavada and Maley [31] evaluated the MT-PCR to look for 12 *β*-lactamases genes in cultured Gram-negative isolates, achieving 95% sensitivity and 96.7% specificity [31].

Singh et al. [32] have developed a real-time multiplex PCR test to detect 10 *β*-lactamases, such as ESBLs, AmpCs, and carbapenemases genes. The diversity of genes sought was higher than in our study, although the *bla_CTX-M 9_* group was neglected [32].

Moreover, Willemsen et al. [33] used qPCR to detect ESBL-encoding genes (*bla_CTX-M-like_*, *bla_TEM_*, and *bla_SHV_*) accessing 98.9% sensitivity and 100% specificity compared to a reference chip [33].

In this study, we also investigated the relationship between phenotypic and genotypic results of ESBL-producing clinical isolates of *E. coli* and *K. pneumoniae*. We detected a relatively high percentage of genes previously shown to be associated with resistance to antibiotics belonging to the *β*-lactams [34].

The strains which carry the SHV and TEM genes show only relatively low resistance to third-generation cephalosporins such as cefixime, cefotaxime, ceftazidime, and monobactam; when coexisting with the genes of the blaCTX-M group, the rate resistance of these bacteria to these antibiotics will be significantly increased [35]. Apart from the many variants of CTX-M that have been reported in recent years, CTX-M-15 belongs to a specific group of these genes, which is defined by increased hydrolysis activity of ceftazidime [36].

Strains with the blaCTX-M-9 gene group only are characterized by a relatively low level of resistance to CAZ, but in combination with blaCTX-M-15, this resistance was markedly increased. The resistance of strains to CTX and CAZ may be explained by the presence of blaCTX-M15 [3].

The blaTEM and blaCTX-M-9 group genes were positively related with resistance to more than four *β*-lactams, according to statistical analysis of our data.

The CMY-2 gene encoded by the plasmid was detected by qPCR in 51.7% of cefoxitin resistant isolates and this result was statistically significant (*P* < 0.05). These results were consistent with two studies conducted in Egypt by Rensing et al. [8] and Fam et al. [37] in which CMY-2 was detected in 86.9% and 76.5%, respectively.

Three of *K. pneumoniae* and one *E. coli* strains carrying *bla_OXA-48_* are resistant to imipenem. *β*-Lactamase OXA-48 hydrolyze significantly carbapenems such as imipenem and penicillins, but not extended-spectrum cephalosporins [38].

These findings support the idea that the qPCR technique can reveal the link between certain *bla* group genes and resistance to multiple *β*-lactam drugs. Multiple resistance genes coexisting in a single strain increase the risk of them spreading to new strains, and the diversity of their resistance complicates molecular detection and treatment.

However, despite the sensitivity of 100% was achieved for resistance tested in clinical urine and culture isolates, the qPCR system could not detect new or currently rare determinants if their number increases over time, which limits the number of targets that can be screened. In addition, this system could not distinguish the genes which code for ESBLs and non-ESBLs from *bla_TEM_* and *bla_SHV_*, as long as they are 10 times rarer than *bla_CTX-M_* among *E. coli* causing urinary tract infections [39].

Thus, our system does not interfere with the collapse antherotherapy, indeed during our work we have used qPCR to detect, only, the variants of ESBL frequently found in our region.

Finally, qPCR cannot predict resistance to cephalosporins and carbapenems in *Enterobacterales* isolates which is caused only by *β*-lactamases, but by other resistance mechanisms such as changes in membrane permeability and efflux pump [40]. These limitations could be linked with those of the conventional method, which only gives results for at least 2 days. If resistance prevails, this shows that most patients are undertreated either by a random treatment, by an agent with limitations but little resistance, or by an antibiotic which would usually be reserved (such as ertapenem) becomes the standard of empirical care.

## 5. Conclusion

In conclusion, the real-time PCR system accurately detected *β*-lactamase-producing *Enterobacterales* directly from biological samples or using purely isolated colonies.

Our results showed a concordance between the results found by the classical method and those by the molecular method. Here, we showed the high prevalence of ESBLs in Tunisia. In summary, an efficient detection system could be put in place to have a diagnosis, a rapid, specific, and reliable antibiotic therapy, and the management of infection control programs. All the tests validated during our work will be soon be marketed as a rapid and cost-effective methods in the laboratory.

## Figures and Tables

**Figure 1:** Distribution of the 7 resistance genes in the 44 *E. coli* and 34 *K. pneumoniae* clinical strains.

**Table 1:** List of primers used for qPCR amplification of ESBLs and carbapenemase genes.

Genes	Primer sequence (5′→3′) FW: Forward RV: Reverse	T°m	Product size (bp)	GenBank
*bla_SHV-12_*	FW: AGCCGCTTGAGCAAATTAAA	59.99	77	LC229232.1
	RV: GCTGGCCAGATCCATTTCTA	60.18		

*bla_TEM_*	FW: GATAAATCTGGAGCCGGTGA	60.04	78	MG860488.1
	RV: GATACGGGAGGGCTTACCAT	60.17		

*bla_CTX-M-15_*	FW: CACCAATGATATTGCGGTGA	60.34	77	MG288677.1
	RV: GTTGCGGCTGGGTAAAATAG	59.61		

*bla_CTX-M-9_*	FW: TACTTCACCCAGCCTCAACC	60.11	78	CP028990.1
	RV: ACCGTCGGTGACGATTTTAG	59.99		

*bla_CMY-2_*	FW: CCAGAACTGACAGGCAAACA	59.87	65	LC229227
	RV: CCTGCCGTATAGGTGGCTAA	60.11		

*bla_OXA-48_*	FW: GTAGTCAGCGCATCGTGAAA	60.02	73	MN654469.1
	RV: CCCGTTTTAGCCCGAATAAT	60.12		

*bla_IMP-1_*	FW: GCCAAAGTCCGCCAAATTAT	60.17	92	MK088089.1
	RV: TCAAGAGTGATGCGTCTCCA	65.56		

*bla_NDM-1_*	FW: ATGGAGACTGGCGACCAAC	61.10	87	LC413788.2
	RV: GGCATGTCGAGATAGGAAGG	59.65		

**Table 2:** Specificity and sensitivity of the qPCR system for *bla* group gene detection.

Resistance gene target	Clinical urines (*n* = 78)					Strains (*n* = 78)				
	True (+) = A	False (-) = B	False (+) = C	True (-) = D	Sensitivity; specificity, %	True (+) = A	False (-) = B	False (+) = C	True (-) = D	Sensitivity; specificity, %
*bla_SHV-12_*	34	0	0	44	100; 100	34	0	0	44	100; 100
*bla_TEM_*	46	0	0	32	100; 100	46	0	0	32	100; 100
*bla_CTX-M15_*	56	0	0	22	100; 100	56	0	0	22	100; 100
*bla_CTX-M9_*	42	0	0	36	100; 100	42	0	0	36	100; 100
*bla_CMY-2_*	29	0	0	49	100; 100	29	0	0	49	100; 100
*bla_OXA-48_*	7	0	0	71	100; 100	7	0	0	71	100; 100
*bla_IMP-1_*	0	0	0	78	100; 100	0	0	0	78	100; 100
*bla_NDM-1_*	1	0	0	77	100; 100	1	0	0	77	100; 100

**Table 3:** The most frequent gene combinations in *E. coli* and *K. pneumoniae* strains.

Genotype	*E. coli*	*K. pneumoniae*
	Number of strains (*n* = 44)	Number of strains (*n* = 36)
*bla_TEM/CTX-M-15/CTX-M-9_*	10	6
*bla_TEM/SHV-12/CMY-2_*	10	7
*bla_SHV-12/CTX-M-15/CTX M-9/TEM_*	5	5
*bla_CMY 2/SHV-12/CTX-M-15/CTX-M-9/TEM_*	2	1

**Table 4:** Antibiotic susceptibility profile of multidrug *E. coli* and *K. pneumoniae.*

Antibiotics	*E. coli* (*n* = 44) (95% CI)		*K. pneumonia*e (*n* = 34) (95% CI)	
	Resistant	Sensitive	Resistant	Sensitive
AMX	100% (44)	0	100%(34)	0
AMC	97.7% (43) [87.99%-99.92%]	2.3% (1)	100%(34)	0
TIC	100% (44)	0	100%(34)	0
CF	100% (44)	0	100%(34)	0
FOX	9.1% (4) [2.53%-21.66%]	90.9% (40) [78.33%-97.46%]	41.2% (14) [24.64%-59.30%]	58.8% (20) [40.69%-75.35%]
CFM	97.7% (43) [87.99%-99.92%]	2.3% (1)	97.1% (33)[84.67%-99.92%]	2.9% (1)
CAZ	97.7% (43) [87.99%-99.92%]	2.3% (1)	94.1% (32) [80.32%-99.27%]	5.9% (2) [0.72%-1.96%]
CTX	97.7% (43) [87.99%-99.92%]	2.3% (1)	97.1% (33) [84.67%-99.92%]	2.9% (1)
IMP	2.3% (1)	97.7%(43) [87.99%-99.92%]	29.4% (10) [15.09%-47.47%]	70.6% (24) [52.52%-84.90%]
AN	25% (11) [13.19%-40.33%]	75% (33) [59.66%-86.80%]	17.6% (6) [6.76%-34.53%]	82.4% (28) [65.46%-93.23%]
GM	45.5% (20) [30.39%-61.15%]	54.5% (24)[38.84%-69.60%]	61.8% (21) [43.56%-77.83%]	38.2% (13) [22.16%-56.43%]
NET	59.1% (26) [43.24%-73.66%]	40.9% (18)[26.33%-56.75%]	52.9% (18) [35.12%-70.22%]	47.1% (16) [29.77%-64.87%]
NN	63.6% (28) [47.77%-77.59%]	36.4% (16)[22.40%-52.2%]	61.8% (21) [43.56%-77.83%]	38.2% (13) [22.16%-56.43%]
NA	88.6% (39) [75.44%-96.20%]	11.4% (5)[11.36%-37.94%]	85.3% (29) [68.94%-95.04%]	14.7% (5) [4.95%-31.05%]
OFX	95.5% (42) [84.52%-99.44%]	4.5% (2)[0.5%-1.54%]	85.3% (29) [68.94%-95.04%]	14.7% (5) [4.95%-31.05%]
CIP	93.2% (41) [81.34%-98.57%]	6.8% (3)[1.42%-18.65%]	82.4% (28) [65.46%-93.23%]	17.6% (6) [6.76%-34.53%]
FFL	9.1% (4) [2.53%-21.66%]	90.9% (40)[78.33%-97.46%]	50% (17) [32.42%-67.57%]	50% (17) [32.42%-67.57%]
SXT	68.2% (30) [52.42%-81.39%]	31.8% (14)[18.60%-47.57%]	67.6% (23)[49.47%-82.61%]	32.4% (11) [17.38%-50.52%]
CL	0	100% (44)	0	100%(34)

AMX: amoxicillin; AMC: amoxicillin + clavulanic acid; TIC; ticarcillin; CF: cephalexin; CFM: cefixime; FOX: cefoxitin; CTX: cefotaxime; CAZ: ceftazidime; IMP: imipenem; NA: nalidixic acid; OFX: ofloxacin; CIP: ciprofloxacin; AN: amikacin, GM: gentamycin; NET: netilmicin; NN: tobramycin; FFL: fosfomycine; SXT: trimethoprim + sulfamide; CL: colistin.

**Table 5:** Correlation between bla genes and antibiotic resistance in the 78 clinical strains (by the *χ*^2^ test).

Antibiotics	*blaTEM*			*blaSHV-12*			*blaCTX-M9*			*blaCTX-M15*			*blaCMY-2*			*blaOXA-48*		
	+	-	*P* value	+	-	*P* value	+	-	*P* value	+	-	*P* value	+	-	*P* value	+	-	*P* value
Resistance to ≥4 *β*-lactam antibiotics	32.60% (15/46)	6.25% (2/32)	0.006	23.52% (8/34)	20.45% (9/44)	0.744	33.33% (14/42)	8.33% (3/36)	0.008	17.85% (10/56)	31.81% (7/22)	0.179	- -	- -	—	66.66% (4/6)	18.05% (13/72)	0.006

**Table 6:** Relationship between bla genes and antibiotic resistance in the 78 clinical strains (by multiple logistic regression analysis).

Antibiotics	Resistance rate % (positive/total)																	
	*blaTEM*			*blaSHV-12*			*blaCTX-M9*			*blaCTX-M15*			*blaCMY-2*			*blaOXA-48*		
	*χ* ^2^	*P* value	OR (95% CI)	*χ* ^2^	*P* value	OR (95% CI)	*χ* ^2^	*P* value	OR (95% CI)	*χ* ^2^	*P* value	OR (95% CI)	*χ* ^2^	*P* value	OR (95% CI)	*χ* ^2^	*P* value	OR (95% CI)
Resistance to ≥4 *β*-lactam antibiotics	5.921	0.015	9.372 (1.545-56.834)	—	—	—	3.764	0.05	4.448 (0.985-20.087)	—	—	—	—	—	—	5.049	0.025	13.100 (1.389-123.552)
FOX	—	—	—	—	—	—	—	—	—	—	—	—	9.835	0.002	11.136 (2.469-50.226)	—	—	—

**Table 7:** Correlation between bla genes and antibiotic resistance in the 78 clinical strains (by Spearman's rank correlation analysis).

Antibiotics	Resistance rate % (positive/total)					
	*blaTEM*	*blaSHV-12*	*blaCTX-M9*	*blaCTX-M15*	*blaCMY-2*	*blaOXA-48*
	*P* value	*P* value	*P* value	*P* value	*P* value	*P* value
Resistance to ≥4 beta-lactam antibiotics	0.002	0.404	0.024	0.264	—	0.002
FOX	—	—	—	—	0.022	0.008

## Data Availability

All data and additional information regarding this study are available to third parties under reasonable request.
